# Levels and Clinical Significance of Regulatory B Cells and T Cells in Acute Myeloid Leukemia

**DOI:** 10.1155/2020/7023168

**Published:** 2020-10-06

**Authors:** Qiaofeng Dong, Guosheng Li, Claudio Fozza, Shuli Wang, Shuhuan Yang, Yuqi Sang, Xinguang Liu, Chunyan Chen

**Affiliations:** ^1^Department of Hematology, Qilu Hospital, Shandong University, Jinan 250012, China; ^2^Department of Hematology, Heze Municipal Hospital, Heze 274000, China; ^3^Blood Diseases Department of Medical, Surgical and Experimental Sciences University of Sassari, Sassari 07100, Italy

## Abstract

Acute myeloid leukemia (AML) is a heterogeneous hematological malignancy, whose immunological mechanisms are still partially uncovered. Regulatory B cells (Bregs) and CD4+ regulatory T cells (Tregs) are subgroups of immunoregulatory cells involved in modulating autoimmunity, inflammation, and transplantation reactions. Herein, by studying the number and function of Breg and Treg cell subsets in patients with AML, we explored their potential role in the pathogenesis of AML. Newly diagnosed AML patients, AML patients in complete remission, and healthy controls were enrolled. Flow cytometry was used to detect percentages of Bregs and Tregs. ELISA was conducted to detect IL-10 and TGF-*β* in plasma. The mRNA levels of IL-10 and Foxp3 were measured with RT-qPCR. The relationship of Bregs and Tregs with the clinicopathological parameters was analyzed. There was a significant reduction in the frequencies of Bregs and an increase of Tregs in newly diagnosed AML patients compared with healthy controls. Meanwhile, patients in complete remission exhibited levels of Bregs and Tregs comparable to healthy controls. Furthermore, compared with healthy controls and AML patients in complete remission, newly diagnosed AML patients had increased plasma IL-10 but reduced TGF-*β*. IL-10 and Foxp3 mRNA levels were upregulated in the newly diagnosed AML patients. However, there were no significant differences in IL-10 and Foxp3 mRNA levels between patients in complete remission and healthy controls. Bregs and Tregs have abnormal distribution in AML patients, suggesting that they might play an important role in regulating immune responses in AML.

## 1. Introduction

Acute myeloid leukemia (AML) is a group of heterogeneous malignant diseases derived from myeloid hematopoietic cells. It is the most common acute leukemia in adults, accounting for about 80% of all adult acute leukemias [1]. Studies have shown that the pathogenesis of AML involves cytogenetic aberrations, acquired mutations, and genetic disorders [2, 3]. Despite advances in the diagnosis and treatment of AML, a significant number of patients have relapses and poor prognosis. Increasing evidence suggests that immune disorders play a key role in the pathogenesis of malignant tumors. Therefore, immunotherapy is a promising strategy for various malignant diseases. For example, the immune escape of tumor cells can be prevented by adjusting immune checkpoints [4–6]. In the past few years, immunotherapy has been increasingly used in the treatment of AML [7, 8]. However, the immune mechanisms and pathways involved in the pathogenesis of AML have only been partially elucidated.

CD4+ regulatory T cells (Tregs) are a subset of T cells that play a role in maintaining self-tolerance and play an important role in the occurrence and development of a variety of malignant diseases including AML [9–11]. Similar to Tregs, regulatory B cells (Bregs) represent a subset of B cells with immunoregulatory properties. They suppress the immune response by producing regulatory cytokines (such as IL-10 and TGF-*β*) and interacting with effector cells (such as effector T cells) [5, 12]. Thus, Bregs play an important role in the pathogenesis of autoimmune diseases, chronic inflammatory diseases, and malignant diseases [13, 14]. However, little is known about the profile of Bregs and Tregs in AML and their possible relationship with AML.

Herein, we investigated the role of Bregs and Tregs in terms of both the number and functions during the course of AML. Our findings may help to elucidate their possible role in the pathogenesis of AML.

## 2. Materials and Methods

### 2.1. Patients

Totally, 40 newly diagnosed (ND) AML patients and 25 AML patients in complete remission (CR) were enrolled from the Department of Hematology, Qilu Hospital, Shandong University, Jinan. The ND AML patients included 18 females and 22 males, with an age range of 21–82 years and a median age of 50 years. There were 12 females and 13 males in AML patients in CR, and their ages ranged from 19 to 71 years, with a median age of 46 years. AML was diagnosed according to the World Health Organization (WHO 2016) classification system. CR was defined based on the International Working Group Criteria. All CR patients except acute promyelocytic leukemia with PML-RARA (APL with PML-RARA) received 3 + 7 standard regimen of anthracycline and cytarabine. APL with PML-RARA patients were treated with both retinoic acid and arsenic trioxide. ND AML patients were not taking any antileukemic therapy at blood sampling. The blood samples of CR patients were collected at 2-3 weeks after the last chemotherapy when patients were in CR. For the control, 15 healthy individuals from the physical examination center of the same hospital were also enrolled, including 10 females and 5 males with an age range of 18–67 years and a median age of 38 years. The basic clinical data of all enrolled subjects are provided in Table 1. Our study was approved by the Medical Ethical Committee of Qilu Hospital, Shandong University. Informed consent was obtained from all participants.

### 2.2. Sample Collection

The EDTA-anticoagulated venous peripheral blood (5 mL) was collected from each subject. Plasma was collected after centrifugation (1500 rpm, 5 minutes) and stored at -40°C until further use. Peripheral blood mononuclear cells (PBMCs) were isolated by density gradient centrifugation using Ficoll separation media (Tianjin Haoyang Biological Manufacture, China).

### 2.3. Flow Cytometric Analysis of Bregs and Tregs

For the detection of Tregs, EDTA-anticoagulated whole blood (100 *μ*L) was stained with FITC-conjugated anti-CD4, PE-conjugated anti-CD25, and APC-conjugated anti-CD127 for 25 minutes at room temperature in the dark. Then, red blood cells were lysed using red blood cell lysis buffer for another 10 minutes. For the detection of Bregs, we used a cocktail of APC-conjugated anti-CD19, PE-conjugated anti-CD24, and FITC-conjugated anti-CD38. All the antibodies were purchased from eBioscience (San Diego, CA, USA). Appropriated species- and isotype-matched IgGs were used as controls. A BD FACSCalibur Flow Cytometer was used. Data were analyzed with Kaluza Flow Cytometry Analysis Software (Beckman Coulter).

### 2.4. Enzyme-Linked Immunosorbent Assay (ELISA)

The levels of IL-10 and TGF-*β* in plasma were measured by ELISA kits following the manufacturer's instructions (eBioscience, San Diego, CA). Briefly, 50 *μ*L of assay buffer was added to each well, and 50 *μ*L of the sample was added within 15 minutes. Then, 100 *μ*L of the detection antibody was added and incubated at room temperature for 2 hours. After washing, 100 *μ*L of the substrate was added and the OD value was detected by a microplate reader. The detection limits of IL-10 and TGF-*β* were 12.95 ng/mL and 108.74 ng/mL, respectively.

### 2.5. RT-PCR

Total RNA was extracted from PBMCs using the TRIzol reagent (Invitrogen, Carlsbad, CA, USA). RNA was reverse transcribed into cDNA using the PrimeScript RT Reagent Kit (Takara Bio Inc., Dalian, China). The reverse transcription reaction procedure was 65°C for 5 minutes, followed by 25°C for 5 minutes, 42°C for 60 minutes, and 70°C for 5 minutes. Real-time PCR was performed on the Applied Biosystems 7500 Real-Time PCR System (Applied Biosystems, Foster City, CA, USA). Each sample was analyzed in triplicate. The primer sequences were shown as follows: IL-10 forward 5′-CTG CCT AAC ATG CTT CGA GA-3′, reverse 5′-CCC TTA AAG TCC TCC AGC AA-3′; Foxp3 forward 5′-TCC CAG AGT TCC ACA AC-3′, reverse 5′-ATT GAG TGT CCG CTG CTT CT-3′; and GAPDH forward 5′-GAA GGT GAA GGT CGG AGT C-3′, reverse 5′-CAT GTA AAC CAT GTA GTT GAG GTC-3′. The levels of target genes were compared to the housekeeping gene GAPDH using the comparative delta Ct (*ΔΔ*Ct) method.

### 2.6. Statistical Analysis

Statistical analyses were performed with SPSS 18.0. All values are expressed as the mean ± SD. For normally distributed data, differences among groups were compared by one-way ANOVA followed by the Student-Newman-Keuls test. Otherwise, the Kruskal-Wallis test followed by the Nemenyi test was used. A *P* value < 0.05 was considered to be of statistical significance.

## 3. Results

### 3.1. Changes of Bregs and Tregs in ND AML Patients and CR Patients

To determine the ratios of Bregs and Tregs in AML patients, flow cytometry was performed. The percentages of Bregs among total CD19+ B lymphocytes were significantly decreased in ND AML patients compared to healthy controls (0.61% ± 0.44% vs. 3.67% ± 1.04%, *P* < 0.001) (Figures 1(a) and 1(b)). Moreover, AML patients in CR had a significantly higher level of Bregs (3.75% ± 1.88%, *P* < 0.001) compared with ND AML patients. Meanwhile, we compared the frequencies of Bregs between AML patients in CR and healthy controls and no difference was observed (*P* > 0.05).

Contrary to Bregs, the percentages of CD4+CD25+CD127- Tregs among CD4+ T cells were higher in ND AML patients (13.77% ± 5.05%), when compared with healthy controls (8.34% ± 1.48%, *P* < 0.001) (Figures 1(c) and 1(d)). A significant decrease of Tregs was also observed in patients in CR (7.09% ± 1.51%, *P* < 0.001) compared with ND patients. However, there were no significant differences in the percentages of Tregs between patients in CR and healthy controls (*P* > 0.05). These results indicate that the abnormal proportion of Bregs and Tregs may be involved in the pathogenesis of AML.

### 3.2. Plasma Levels of IL-10 and TGF-*β*

We further examined the concentrations of IL-10 and TGF-*β* in plasma by ELISA. Compared with healthy controls (*n* = 15) and AML patients in CR (*n* = 25), ND AML patients (*n* = 40) had significantly higher plasma IL-10 (*H* = 6.98, *P* = 0.03). However, there was no significant difference in plasma IL-10 between CR patients and healthy controls (Figure 2(a)). On the contrary, the concentration of TGF-*β* was lower in ND AML patients, compared with healthy controls and AML patients in CR (*H* = 10.95, *P* = 0.004) (Figure 2(b)). And no significant differences were found between patients in CR and healthy controls.

### 3.3. IL-10 and Foxp3 Are Upregulated in ND AML Patients

Then, we determined IL-10 and Foxp3 mRNA levels by RT-PCR in human PBMCs. As shown in Figure 3(a), IL-10 was increased in ND AML patients (*n* = 40) compared with healthy controls (*n* = 15) and patients in CR (*n* = 25) (*H* = 21.24, *P* < 0.001). The expression of Foxp3 mRNA was also upregulated in ND AML patients compared with healthy controls (*P* < 0.001) and AML patients in CR (*P* < 0.001) (Figure 3(b)). Moreover, there were no significant differences in IL-10 and Foxp3 mRNA levels between patients in CR and healthy controls.

## 4. Discussion

T cells and B cells are involved in cellular and humoral immunity and play a pivotal role in immune surveillance against malignant clones. Among them, Tregs and Bregs are cell subgroups displaying specific immune regulatory properties in preventing excessive immune responses. It has been reported that Tregs and Bregs could repress autoimmunity and inflammation and facilitate tumor progression [14, 15]. Studies have shown that elevated percentages and enhanced functions of Tregs contribute to a variety of malignancies [9, 14, 16, 17], including AML [18].

However, little is known about the profile of peripheral Bregs in AML patients. In the present study, based on the previous description [19], Bregs were identified as CD19+CD24hiCD38hi cells. Our results showed that the percentages of Bregs were significantly reduced in ND AML patients compared with healthy controls. Breg levels recovered to normal levels in patients with CR, suggesting that Breg plays a possible role in the pathogenesis of AML. IL-10 and TGF-*β* are key modulators in immune tolerance and in regulating the functions of Bregs and Tregs [20]. In our study, we observed increased plasma IL-10 and decreased TGF-*β* levels in ND AML patients, suggesting the disturbed immune homeostasis in these patients. Bregs and Tregs could secret both IL-10 and TGF-*β* [21, 22]. However, other cell types such as monocytes/macrophages, and dendritic cells are also able to produce IL-10 and TGF-*β* [23–25]. Karim et al. [26] reported that CD19+CD24+CD38hi Bregs may be a small subset within a large population of IL-10-producing B cells, which on the whole are only identifiable by their capability to express IL-10. Our results suggested that Bregs and Tregs may participate in the dysregulation of immune responses and cytokine secretion in AML.

The number and functions of Tregs are reported to be enhanced in some solid tumors, facilitating the immune escape [17, 27]. Consistently, our data showed that the percentages of Tregs were higher in ND AML patients compared with healthy controls and AML patients in CR. Furthermore, ND AML patients had higher mRNA expression of Foxp3 compared to AML patients in CR and healthy controls.

Bregs have been found to suppress the proliferation of CD4+ T cells and enhance Foxp3 and CTLA-4 expression in Tregs [28]. Accumulating evidence has shown the interaction between Bregs and Tregs in the cancer microenvironment [5, 15, 22]. It is reported that the decreased frequencies of peripheral Tregs or increased frequencies of Bregs might be modulated directly by lung cancer cells [5]. Bregs in the context of breast cancer could induce the conversion of resting CD4+ T cells to Tregs to facilitate the lung metastasis [15]. In addition, cytokines including IL-12, IFN-*γ*, and IL-21 strictly regulate the production of IL-10 by B cells and the above cytokines specifically regulate the development and activity of Tregs and IL-10-producing Bregs [22]. Thus, we suppose that the abnormal distributions of Bregs and Tregs might be regulated by several cytokines, which are aberrant in ND AML and restored after CR. Tumor recurrence and metastasis are potentially promoted by the impairment of immune surveillance mechanisms [28].

Conventional cancer therapies, such as chemotherapy, radiation therapy, and even targeted therapy, are only partially able to control neoplastic clones. Treatments based on immunotherapy are now widely applied to AML with satisfactory outcomes [29, 30]. Treatment involving Treg modulation has been proposed to enhance anticancer immunity [31]. Bregs may also be identified as new potential beneficial targets to improve the prognosis of AML patients.

## 5. Conclusions

We reported the levels of both peripheral Tregs and Bregs in a cohort of AML patients. Bregs were decreased in ND AML patients and recovered after achieving CR, whereas Tregs were elevated in ND AML patients and reduced in CR. These results indicate the abnormal distribution of these cell subsets in AML patients and suggest that a postchemotherapy combined strategy targeting Tregs and Bregs could be potentially beneficial for the management of AML patients in the future.

## Figures and Tables

**Figure 1:** Frequencies of peripheral Bregs and Tregs were detected in normal controls, ND AML patients, and AML patients in CR. (a) Representative flow cytometry analysis of peripheral CD19+CD24hiCD38hi Breg populations. (b) Frequencies of Bregs among CD19+ B cells in different groups. (c) Representative dot plot of peripheral CD4+CD25+CD127- Treg populations. (d) Frequencies of Tregs in CD4+ T cells in different groups. ^∗∗∗^*P* < 0.001. *n* = 15, 40, and 25, respectively.

**Figure 2:** The levels of IL-10 and TGF-*β* in healthy controls, ND AML patients, and AML patients in CR by ELISA. (a) Concentrations of IL-10 in different groups. (b) Concentrations of TGF-*β* in different groups. ^∗^*P* < 0.05, ^∗∗^*P* < 0.01.

**Figure 3:** Analysis of IL-10 and Foxp3 mRNA expression by RT-qPCR. (a) IL-10 mRNA expression was elevated in ND AML patients compared with healthy controls and AML patients in CR. (b) Significantly higher levels of Foxp3 mRNA expression were observed in ND AML patients than in healthy controls or AML patients in CR. ^∗∗^*P* < 0.01, ^∗∗∗^*P* < 0.001.

**Table 1:** The clinical information of all enrolled subjects.

Clinical characteristics	ND AML patients (*n* = 40)	CR AML patients (*n* = 25)	Controls (*n* = 15)
Age (years, median, range)	50 (21–82)	46 (19–71)	38 (18–67)
Sex (male/female)	22/18	13/12	5/10
WBC (×10^9^/L)	40.51 ± 48.67	4.60 ± 2.50	4.50 ± 2.70
HGB (g/L)	68.79 ± 23.57	120.12 ± 26.44	120.31 ± 18.34
PLT (×10^9^/L)	59.94 ± 68.48	205.25 ± 120.15	245.25 ± 130.65
BM leukemic blasts (%)	76.81 ± 19.52	1.89 ± 0.78	—
Abnormal karyotype (*n*, %)	24 (60%)	4 (16%)	—
WHO (2016) classification			
Acute myeloid leukemia with recurrent genetic abnormalities	13	15	—
Acute myeloid leukemia with myelodysplasia-related changes	2	1	—
Therapy-related myeloid neoplasms	1	0	—
AML, not otherwise specified	24	9	—

Note: AML: acute myeloid leukemia; ND: newly diagnosed; CR: complete remission; WBC: white blood cells; HGB: hemoglobin; PLT: blood platelet; BM: bone marrow.

## Data Availability

The data that support the findings of this study are available on request from the corresponding authors.
